# A Public Health-Oriented New Energy Industry Competitiveness Evaluation

This article has been retracted.

**DOI:** 10.1155/2022/4573629

**Published:** 2022-08-18

**Authors:** Zhijie Dou, Li Shi Li, Lu Lu

**Affiliations:** ^1^School of Management, Changchun University, Changchun 130022, China; ^2^Shenzhen Xhorse Electronics Co., Ltd, Shenzhen 518000, China

## Abstract

This paper develops a regional new energy industry (NEI) competitiveness evaluation index system based on the theoretical framework of the “diamond model” and the unique characteristics of the new energy industry and made an empirical analysis of Jilin province with analytic hierarchy process (AHP) and fuzzy comprehensive evaluation method. The analysis results show that the new energy industry in Jilin Province has a good foundation, and the government's role, talent support, technological innovation, and market factors are acceptable. However, due to location factors and resource endowments, regional GDP and per capita consumption expenditure are low. The lack of intrinsic motivation of industrial competitive advantage has resulted in the poor overall competitiveness of the new energy industry in Jilin Province. Then, it is advised to take targeted measures to work closely with national NEI development strategy, optimize the industrial technology innovation ability and the talent support, actively guide social capital flows and new energy consumption, optimize regional energy consumption structure and industrial structure by creating a complete NEI chain, and revitalize the whole economy.

## 1. Introduction

The meaning of “public health” refers to the science and technology that examines social groupings with the goal of preventing disease, increasing life expectancy, and protecting people's health. To guide, promote, and preserve human health, it is a mix of scientific knowledge, practical skills, and religious beliefs. The progress of social groupings in concert with one another is necessary for the achievement of public health goals. In recent years, the improper use of traditional forms of energy has resulted in damage to the environment as well as issues with public health. In particular, energy consumption that is based on fossil fuels, such as the burning of coal, produces a wide variety of pollutants into the atmosphere, some of which include SO2, soot, PM, and NOx. They contribute to the deterioration of air quality, cause and exacerbate a variety of health hazards, including respiratory disorders, cardiovascular diseases, and lung cancer, and even the sudden death of sensitive populations, which poses a significant risk to the general population's health [1,2]. According to reference [3], greenhouse gas emissions are the primary factors contributing to the deterioration of the ecosystem. Through the use of the investigative report, Edwin Chadwick established a compelling case that the issue with public health is more closely related to environmental issues than it is to medical issues [4]. The first version of “the Public Health Act” [5] was enacted in the United Kingdom. This act stipulated the form of buildings and streets from the perspective of environmental sanitation. Additionally, it stipulated the requirements for urban sewage discharge and garbage transfer. From 2010 to 2030, the yearly rate of growth in the use of energy across the globe is projected to be 1.7% [6,7]. As a result, it is of the utmost significance to work toward the improvement of public health from the point of view of the expansion of the new energy business.

The generation of new energy is essential to the accomplishment of sustainable development since it is intertwined with social, economic, and environmental progress. Participation from members of the general population is required for the discovery of new energy sources [8,9]. Understanding the competitiveness of the NEI in Jilin Province is essential for determining the limiting factors, optimizing the regional energy consumption structure and industrial structure, and increasing the overall competitiveness of the regional economy. This can be accomplished by conducting an accurate and scientific evaluation of the competitiveness level of the NEI in Jilin Province.

## 2. Relevant Knowledge

### 2.1. Connotation of Industrial Competitiveness

An enterprise is said to have an industrial competitive advantage if it is able to achieve cheap costs and high profit in a particular market as a result of its business activity system, which is difficult to copy or imitate by the enterprise's other competitors. Because of this, industrial competitiveness can also be thought of as a form of comparative productivity. In terms of its breadth, the concept of industrial competitiveness can be broken down into two categories: regional and localism. It is possible to draw comparisons from a relatively wide range of fields and scopes. Comparisons can be made across multiple countries or areas, or they can be made internally within the same country or territory. Either way, they can be useful. The level of industrial competitiveness can be seen reflected not only in the differences between explicit indicators like industrial level, industrial scale, and market share, but also in the differences between implicit indicators like input factors, industrial environment, and technological level. Explicit indicators include things like industrial level, industrial scale, and market share. Implicit indicators include things like input factors, industrial environment, and technological level. The most important ones among them are the ones that accurately reflect the common sense findings regarding the level of industrial competitiveness in the region. Indicators that are trending downward are almost always the primary factor that underlies a decline in the competitiveness of regional sectors. In order for the industrial competitiveness evaluation index system to be constructed and evaluated correctly, the following principles—namely, the scientific principle, the feasibility principle, and the combination principle of process index and state index—need to be adhered to.

### 2.2. The Particularity of the New Energy Industry

Energy demand and use affect all aspects of the natural and social environment, and affordable and reliable energy is critical to meeting basic human needs and can be a cornerstone of development [10,11]. New energy industry development is a critical strategy and means for China to implement sustainable development and adjust its industrial structure [12]. New energy is the energy that is distinct from traditional and conventional energy. Solar energy, wind energy, geothermal energy, biomass energy, water energy, and ocean energy are examples of renewable energy sources, as are clean energy and green energy [13]. The NEI refers to a series of processes for the development and utilization of new energy carried out by units or enterprises.

Agriculture, industry, and consumer spending are the three primary areas that are traversed by the supply chain of the NEI as it moves from point A to point B. There are a significant number of links or departments in the industrial chain due to the fact that the majority of the subsequent processing steps take place in the industrial sector. Despite this, the relationship between the upstream and downstream parts of the industrial chain is quite robust. The new energy industry (NEI) is being increasingly impacted and dominated by the industry, as a result of the intensity of the substitution of new energy for the initial energy. Additionally, items in all parts of the NEI participate in significant import and export trade, and the industry is heavily dependent on the worldwide market. This results in increased levels of both uncertainty and risk associated with the industry's future development.

Researchers examine the NEI from the points of view of resources, markets, technologies, and industrial policy. The development of biomass energy in Jilin Province is analyzed and evaluated in reference [14], which uses the reserve, availability, and utilization index l as its primary metrics. The evaluation and research on the competitiveness of Hebei's NEI that is presented in reference [15] takes into account six different factors: the foundation, technology, manpower, economics, environment, and market. The findings of a key success factor analysis are used in the construction of an evaluation system for the wind energy business in Inner Mongolia that is cited in reference [16].

## 3. NEI Competitiveness Evaluation Index System

The article referred to in reference [17] investigates the question of whether or not the government ought to be involved in the adjustment of the energy structure and the future development direction of the energy industry. This investigation is based on the evolutionary game theory. In this paper, the cooperative and competitive relationships that exist in the energy business between the old energy industry and the new energy industry are investigated, and the elements that influence the evolutionary equilibrium strategy are spoken about. A game model was built based on reference [18], which was based on the progression of competitive entities and the market environment. The model runs numerical simulations and investigates in great detail the underlying reasoning behind the behavior choices made by both of the competing groups in the game. The findings of this research offer the government with a theoretical basis on which to base realistic NEI development policies. According to reference [19], the NEI is considered to be a complex system, and the method of system dynamics is utilized in order to model and evaluate it. In conclusion, synergy theory is applied to the dynamic model, and important recommendations for the growth of my country's new energy industry are offered as a result.

In a nutshell, my nation is now conducting a significant number of studies on the NEI. The vast bulk of these studies are devoted to examining how different policies and approaches to business are implemented by various governments. But there have not been many studies conducted on the NEI from the point of view of how it affects industrial competitiveness. The study of industrial competitiveness has a lengthy history, and over that time, a standardized research paradigm as well as a research framework have been developed. This work proposes and builds a regional NEI competitiveness evaluation index system based on the diamond model proposed by American economist Michael Porter. The system is designed to evaluate a region's level of competitiveness relative to other regions.

### 3.1. Theoretical Basis

The “diamond model” developed by Michael E. Porter breaks the industrial competitive advantage of a nation down into four fundamental aspects and two supplementary elements. One of these conditions is known as the factor condition, and it describes the input that must be present in order to manufacture a specific product. This can include things like human resources, natural resources, scientific and technological expertise and so on. The creative process, rather than the availability of resources, is the focal point of this discussion. The second factor is the demand situation, which refers to the amount as well as the quality of the market demand for a specific product or service within an industry. In most cases, the industry's competitive edge is directly impacted by the degree of difficulty of the demand as well as the rate of its development. The third category is comprised of related sectors as well as supporting industries, and it mostly refers to the level of collaboration that exists between upstream and downstream companies. The corporate strategy, organizational structure, and the competition come in at number four. The fifth factor is opportunity, which refers to the chances presented to businesses and industries as a result of changes in the surrounding environment that are beyond their control, such as scientific and technological breakthroughs, natural disasters, and social changes, all of which have the potential to alter the competitive situation that is currently in place. The sixth component is the effect that government action has, either positively or negatively, on the previous four factors through the implementation of industrial policies [20,21]. Later academics made additions to this model that were based on it in order to make it more useful. In 1993, the British academic Dunning included the component of “commercial activities of multinational organizations” to establish a “Porter-Dunning model” that was more comprehensive [22]. When Lugman and Cruz investigated Canada's competitive edge, they combined the Canadian diamond model and the American diamond model to create a double-diamond model [23]. This model combines the advantages of both countries' diamond models. A professor at Seoul University in South Korea named Zhao Dongcheng came up with the idea for a nine-element model based on the current circumstances in South Korea [24].

According to the theoretical framework of the “Diamond Model” and the specificity of the new energy industry, the comprehensive evaluation index system for the competitiveness of the NEI constructed in this paper primarily includes industrial foundation, government role, location factors and resource endowments, technological innovation, talent support, and market factors.  Figure 1 shows basic framework for evaluating the competitiveness of the new energy industry [25]. These six parts are interconnected and mutually reinforcing to form a complete diamond system. This system has the potential to significantly boost the competitiveness of the regional new energy industry.

### 3.2. System Composition

According to the above theoretical analysis framework, this paper proposes the regional NEI competitiveness evaluation index system shown in Table 1. Three layers make up the system: the target layer at the top, which is used to evaluate the level of competitiveness of the regional new energy industry. The element layer, which contains the six basic elements mentioned above, is the second layer. The third layer is the indicator layer, which contains a total of 28 indicators.

The location and resource endowment factors are mainly considered from the six aspects of regional new energy reserves, regional GDP, per capita consumption expenditure, energy production structure, energy consumption structure, and resource abundance.

The industrial foundation: the development foundation of the new energy industry is very important to its competitiveness. It can be reflected in terms of the average fixed assets of the industry, the quality and specifications of industry employees, and the integrity of the industry chain.

Technological innovation: technological innovation is a key factor affecting the development of the new energy industry, which can be reflected by four indicators: R&D capital investment, R&D personnel ratio, independent invention patent ownership rate, and technological competitiveness.

Talent support is measured in terms of human resource investment, the number of colleges and universities, the number of scientific research platforms, and residents' public health awareness and participation.

The role of the government is mainly reflected in four aspects: the strength of policy support, the degree of perfection of the policy system, the capacity of policy supply, and the capacity of restraint.

Market factors mainly consider the strength of policy support, the degree of perfection of the policy system, the capacity of policy supply, and the capacity of policy restraint.

## 4. Empirical Analysis of the Competitiveness Evaluation of NEI

### 4.1. Selection of Evaluation Methods

1. *Analytic Hierarchy Process (AHP).* Reference [26] proposes AHP as a systematic analysis method, which divides the various influencing factors in complex problems correspondingly to form an interconnected and organized orderly hierarchy. AHP analyzes and processes people's subjective judgments using mathematical theory, and it combines quantitative and qualitative analysis to eliminate bias [27]. It compares each hierarchical element pairwise, and describes its importance quantitatively. Then by calculating the order weight, it sorts all the hierarchical factors, and calculates the relative weight of all factors. AHP is generally used for weighted analysis of multiple indicators, and then evaluates the advantages and disadvantages of each scheme under multiple influencing factors. When the decision is affected by multiple factors, and there is a hierarchical relationship between each factor, the AHP method can be used. According to the theory of industrial competitiveness, there are many factors affecting the competitiveness of the new energy industry, and the selection of evaluation indicators is multi-level and hierarchical. Therefore, this method is suitable for selection.
2. *Fuzzy Comprehensive Evaluation (FCE).* It is a comprehensive evaluation method that employs fuzzy mathematics' membership degree theory to convert qualitative evaluation into quantitative evaluation [28]. This evaluation method distinguishes itself by evaluating each object individually. Each evaluation object has a unique evaluation value that is unaffected by the collection in which it is located [29, 30]. It produces results that are both clear and systematic. It can better solve the problems affected by various factors and is suitable for the analysis and processing of various nondeterministic problems. This method provides a better tool for qualitative question evaluation and can reflect the evaluation results more objectively. Although it was proposed late, it has been well used in many fields such as agriculture, information control, and artificial intelligence. The new energy sector is a strategically important emerging sector with a modest total size and challenging data collecting. On the basis of the index system and weights created by the AHP, the fuzzy comprehensive evaluation model will be used in this study to assess the competitiveness of the new energy sector in Jilin Province.

### 4.2. Evaluation Process and Results

#### 4.2.1. Building the Judgment Matrix

The judgment matrix must be built by comparing the relative importance of the indicators in pairs using the analytic hierarchy procedure.  Table 2 displays the important comparison. This study applies the Delphi technique to the process of creating the judgment matrix. The number of experts in the expert group is 9, and the experts are from academic fields, leaders, and managers of related enterprises. Through the introduction of the research and the reading of relevant materials, 9 experts evaluated the relative importance of each indicator.

#### 4.2.2. Test of Relative Weight's Constancy

After three rounds of result statistics, information feedback, and re-discussion, the first-level index judgment matrix shown in Table 3 is finally determined.

After determining the weight distribution of the first-level indicators, formula *CI*=(*λ*_max−*n*_)/(*n* − 1) is used for consistency check to determine whether the weight is reasonable. After calculation, *λ*_max_ = 6.5743, CI = 0.11486, and CR = 0.0912 < 0.1. It conforms to the consistency test, and the weight distribution is reasonable. Using the same calculation process, the judgment matrix of each secondary index (indicator layer) can be calculated, and the consistency test results show that the weight distribution is reasonable.

#### 4.2.3. Judgment Matrix Combined Weight and Consistency Test

Finally, the consistency test of the index layer to the element layer is carried out, CI = 0.02563, RI = 0.40919, CR = CI/RI = 0.02563/0.40919 = 0.06264 < 0.1. Through all levels of inspection, all judgment matrices meet satisfactory consistency. The weight distribution of the indicators at all levels determined in this paper is valid. Overall, the weight distribution of the evaluation index system can better reflect the difference between the NEI and general industries, and can truly and objectively evaluate the competitiveness of strategic emerging industries.

#### 4.2.4. Analysis of Influencing Factors of NEI in Jilin Province

It can be seen from Table 4 that in the ranking of the weights of decision-making objectives at the factor level, technological innovation takes the first place, with a weight of 0.4372. Compared with other peer indicators, its importance is far ahead. This demonstrates that the most important factor limiting the competitiveness of the NEI in Jilin Province is the level of technological innovation. The role of the government ranks second with a weight of 0.199. This indicates the larger role played by the government in the growth of the new energy sector. At the same time, it also proves the necessity of further strengthening and optimizing government control measures in the process of NEI development. The third is talent support, which is in line with the general characteristics of strategic emerging industries. Increasing talent training and investment is the key to rapidly enhancing the competitiveness of the industry. The sum of the weights of the top three indicators accounts for 77.42% of all indicators in the middle layer for decision-making goals. This shows that technological innovation, government role, and talent support are the key factors that determine the overall competitiveness of the NEI in Jilin Province.

By sorting the weights of decision-making targets at the index level (see Figure 2), it is found that the top three are independent invention patent ownership rate, R&D capital investment, and technological competitiveness, with weights of 0.1876, 0.1317, and 0.075, respectively. The sum of the proportions of the three is 0.3943, which once again shows that technological innovation is the primary source of competitiveness of the regional new energy industry. The weight of policy supply capacity is 0.0716, and the weight of human resources investment is 0.0692, ranking the fourth and fifth, respectively. This shows that increasing the talent support and the role of the government in the field of new energy, and focusing on guiding and tapping the market demand for new energy products are also directions to improve the competitiveness of the new energy industry in Jilin Province.

#### 4.2.5. A Fuzzy Comprehensive Evaluation of the NEI's Competitiveness in Jilin Province

According to the constructed index system, a fuzzy comprehensive questionnaire was designed. Rating scale = {V1, V2, V3, V4} = {very good, better, fair, poor} = {4, 3, 2, 1}. Using yaahp analysis software, the collected expert scoring data are processed to obtain the scores of the criterion layer and the index layer. The final score of the fuzzy comprehensive evaluation of the competitiveness of the new energy industry in Jilin Province is 2.4995 points, which belongs to the “general” level. The specific scores are shown in Table 5.

In the fuzzy comprehensive evaluation score of the factor layer, the industrial base has the highest score. It reflects the solid foundation of the new energy industry in Jilin Province, with rich varieties and reserves. Talent support and market factor scores are ranked 2nd and 3rd. On the one hand, it shows that Jilin Province attaches great importance to new energy talents, has accumulated a certain amount of talents who are conducive to the development of the new energy industry, and has a good foundation for industrial development. On the other hand, it shows that the market is active, and the existing market factors in Jilin Province have a greater role in promoting the new energy industry. The lowest score on location factor and resource endowment shows the disadvantage of location factor and resource endowment, which lowers the overall competitiveness score to a large extent.

In the fuzzy comprehensive evaluation score of the index layer, the degree of perfection of the policy system, government restraint ability, demand growth potential, industrial market concentration, resource allocation ability, market growth ability, new energy reserves, resource abundance, industry average fixed assets, the quality and specifications of industrial employees, the integrity of industrial chain development, R&D capital investment, human resource investment, the number of colleges and universities, the number of scientific research platforms, and the degree of residents' public health participation are all at a “good” level. It shows that most of the level of the development of new energy industry in Jilin Province is still acceptable. We should continue to increase investment in these areas, and these indicators are also expected to develop from a “better” level to a “very good” level, and the overall competitiveness level may be improved. The regional GPD and per capita consumption expenditure scores are both “poor” grades, which have become the main indicators that drag down the overall competitiveness.

## 5. Conclusions and Recommendations

This paper develops a regional NEI competitiveness evaluation index system based on the diamond model. Sixteen indicators are chosen to reflect the regional NEI's competitiveness from six categories: location factor and resource endowment, industrial base, technological innovation, talent support, market factor, and government role. Through professional consultation and weight calculation of AHP, it is found that technological innovation and government role are the primary factors affecting the competitiveness of Jilin Province's new energy industry. Increasing talent support and tapping market demand are the main directions for improving the competitiveness of Jilin Province's new energy industry. The specific operation suggestions are as follows:

1. Improve technological innovation capabilities. Increase R&D investment, clarify R&D investment intensity and priority order of the new energy industry, and prioritize scientific and technological innovation. The technology research and development capabilities of enterprises, universities, research institutes, and other units will be integrated through the implementation of major scientific and technological special projects in the new energy industry. We must take on the fundamental technologies of the new energy industry. To reduce production costs and improve safety, focus on breakthroughs in core technologies such as solar energy technology, water energy technology, wind energy technology, biomass energy technology, and so on. To prioritize energy industry development, we must first confront the market, seek maximum benefits, and accelerate the development of the NEI in Jilin Province.
2. Give the government's guiding role a chance. The NEI's foundation should be policy-oriented. The NEI must shoulder the strategic responsibility of environmental governance and energy transformation. The industry as a whole must closely grasp the policy trends and make predictions in advance. The national NEI development strategy should be actively implemented. Formulating more comprehensive, targeted, and promoting NEI development policies in conjunction with the development foundation and development status of Jilin Province. The Jilin provincial government should invest heavily in financial subsidies, particularly in the early stages of NEI cultivation, to ensure adequate development conditions. On the other hand, businesses should pay attention to this issue as well, and ensure the reasonable use of subsidies within the scope of legal norms while ensuring the policy dividends. Make a reasonable development plan, reduce the dependence on government subsidies as soon as possible, and rely on the enterprise's own business behavior to make profits.
3. Strengthen the support of talents. The rational allocation and utilization of talents is an important part of the good development of new energy enterprises. The NEI in Jilin Province should establish a sound recruitment and training mechanism and provide outstanding talents for sales, supply chain, and R&D direction. Jilin Province has high-quality educational resources, a total of 66 colleges and universities, and many colleges and universities have carried out professional courses related to new energy. Enterprises should accept fresh graduates in an appropriate environment, absorb fresh blood, and train highly professional students to undertake R&D, manufacturing, and other related businesses as soon as possible. At the same time, we must attach importance to R&D strength and pay attention to protecting intellectual property rights in competition. Talent support and development need to establish a reasonable assessment and salary adjustment mechanism for different business directions, build a perfect reward and punishment system, and fully combine the two characteristics of new energy: technology-intensive and labor-intensive.

In short, Jilin Province should increase the publicity of new energy products and encourage social capital to enter. The development and layout of the NEI should be combined with the optimization and adjustment of the regional industrial structure by continuously improving the integrity of the development of the NEI chain. Through the aforementioned channels, the NEI can play a larger role in promoting Jilin Province's regional economic revitalization.

## Figures and Tables

**Figure 1:** Basic framework for evaluating the competitiveness of the new energy industry.

**Figure 2:** The ranking weight of the decision target at the indicator layer.

**Table 1:** Competitiveness evaluation index system of NEI in Jilin Province.

Target layer	Feature layer	Indicator layer
Regional NEI competitiveness (A)	Government role (B1)	Policy support strength (C1)
		The degree of perfection of the policy system (C2)
		Policy supply capability (C3)
		Government binding capacity (C4)
	Market factors (B2)	Market share (C5)
		Growth potential of demand (C6)
		Existing firm size (C7)
		Industry market concentration (C8)
		Configure resource capability (C9)
		Market growth capability (C10)
	Location factors and resource endowments (B3)	New energy reserves (C11)
		Regional GDP (C12)
		Per capita consumption expenditure (C13)
		Energy production structure (C14)
		Energy consumption structure (C15)
		Resource abundance (C16)
	Industrial foundation (B4)	Industry average fixed assets (C17)
		Industrial practitioner quality and specifications (C18)
		Completeness of industrial chain development (C19)
	Technological innovation (B5)	R&D capital investment (C20)
		R&D personnel ratio (C21)
		Own invention patent ownership rate (C22)
		Technology competitiveness (C23)
	Talent support (B6)	Human resource input (C24)
		Number of institutions of higher learning (C25)
		Number of scientific research platforms (C26)
		Residents' public health awareness (C27)
		Residents' public health participation degree (C28)

**Table 2:** Importance comparison scale table.

Scale value meaning	Scale value
Both *a* and *b* are equally significant	1
*a* is marginally more important than *b*	3
*a* is more significant than *b*	5
*a* is more significant than *b*	7
*a* is unquestionably more important than *b*	9
The average of two adjacent judgments	2, 4, 6, 8

**Table 3:** Judgment matrix *X* of primary indicators.

A	B1	B2	B3	B4	B5	B6	Wi
B1	1	4	3	2	1/3	2	0.1990
B2	1/4	1	4	2	1/7	1/2	0.0955
B3	1/3	1/4	1	1/3	1/5	1/3	0.0452
B4	1/2	1/2	3	1	1/3	1/3	0.0851
B5	3	7	5	3	1	5	0.4372
B6	1/2	2	3	3	1/5	1	0.1380

**Table 4:** Weight distribution of various indicators in the competitiveness evaluation of NEI in Jilin Province.

	The first dimension (feature layer)	Weights	The second dimension (indicator layer)	Weights
Jilin Province NEI competitiveness evaluation index system	Government role	0.1990	Policy support strength	0.0395
			The degree of perfection of the policy system	0.0567
			Policy supply capability	0.0716
			Government binding capacity	0.0395
	Market factors	0.0955	Market share	0.0085
			Growth potential of demand	0.0402
			Existing firm size	0.0154
			Industry market concentration	0.0041
			Configure resource capability	0.0145
			Market growth capability	0.0128
	Location factors and resource endowments	0.0452	New energy reserves	0.003
			Regional GDP	0.0038
			Per capita consumption expenditure	0.0153
			Energy production structure	0.0039
			Energy consumption structure	0.009
			Resource abundance	0.0101
	Industrial foundation	0.0851	Industry average fixed assets	0.0119
			Quality and specifications of industrial practitioners	0.0449
			Completeness of industrial chain development	0.0283
	Technological innovation	0.4372	R&D capital investment	0.1317
			R&D personnel ratio	0.0428
			Own invention patent ownership rate	0.1876
			Technology competitiveness	0.075
	Talent support	0.1380	Human resource input	0.0692
			Number of institutions of higher learning	0.0077
			Number of scientific research platforms	0.0171
			Residents' public health awareness	0.017
			Residents' public health participation degree	0.0269

**Table 5:** Fuzzy comprehensive evaluation scores of new energy competitiveness in Jilin Province.

	Feature layer	Score	Indicator layer	Score
Jilin NEI competitiveness (A)	Government role (B1)	2.4833	Policy support strength (C1)	2
			The degree of perfection of the policy system (C2)	3
			Policy supply capability (C3)	2
			Government binding capacity (C4)	3
	Market factors (B2)	2.7493	Market share (C5)	2
			Growth potential of demand (C6)	3
			Existing firm size (C7)	2
			Industry market concentration (C8)	3
			Configure resource capability (C9)	3
			Market growth capability (C10)	3
	Location factors and resource endowments (B3)	1.8665	New energy reserves (C11)	3
			Regional GDP (C12)	1
			Per capita consumption expenditure (C13)	1
			Energy production structure (C14)	2
			Energy consumption structure (C15)	2
			Resource abundance (C16)	3
	Industrial foundation (B4)	3.0000	Industry average fixed assets (C17)	3
			Industrial practitioner quality and specifications (C18)	3
			Completeness of industrial chain development (C19)	3
	Technological innovation (B5)	2.3012	R&D capital investment (C20)	3
			R&D personnel ratio (C21)	2
			Own invention patent ownership rate (C22)	2
			Technology competitiveness (C23)	2
	Talent support (B6)	2.8771	Human resource input (C24)	3
			Number of institutions of higher learning (C25)	3
			Number of scientific research platforms (C26)	3
			Residents' public health awareness (C27)	2
			Residents' public health participation degree (C28)	3

## Data Availability

The labeled dataset used to support the findings of this study are available from the corresponding author upon request.
